# The Potential of miR-370-3p and miR-495-3p Serving as Biomarkers for Sepsis-Associated Acute Kidney Injury

**DOI:** 10.1155/2022/2439509

**Published:** 2022-07-11

**Authors:** Wenlu Ma, Xiaomei Miao, Fangfang Xia, Chao Ruan, Dan Tao, Bing Li

**Affiliations:** Department of Nephrology, SINOPHARM North Hospital, Baotou, 014030 Inner Mongolia, China

## Abstract

**Objective:**

This study is aimed at evaluating the miR-370-3p and miR-495-3p expression in the urine of patients with sepsis-associated acute kidney injury (SA-AKI) and exploring its diagnosis value in for SA-AKI.

**Methods:**

184 sepsis invalids were collected and divided two groups (non-AKI group or AKI group) according to whether they had acute kidney injury. RT-qPCR was utilized to measure miR-370-3p and miR-495-3p expressions. ROC curve was performed to evaluate the diagnostic value of miR-370-3p and miR-495-3p for SA-AKI. Patients diagnosed with SA-AKI were followed up for 28 days to record survival time. The prognostic performance of miR-370-3p and miR-495-3p for SA-AKI was evaluated by survival curves.

**Results:**

Compared with non-AKI invalids, miR-370-3p and miR-495-3p expressions were obviously lower in the urine of AKI invalids. miR-370-3p and miR-495-3p expressions were markedly negatively correlated with biomarkers of renal injury. Furthermore, the area under the curve (AUC) of miR-370-3p and miR-495-3p for diagnosing sepsis SA-AKI was 0.896 and 0.814, respectively. The higher 28 days-survival rate was observed in patients with high miR-370-3p and miR-495-3p expressions.

**Conclusions:**

A novel biomarker for the early diagnosis of SA-AKI may be miR-370-3p and miR-495-3p, which was clearly reduced in the urine of SA-AKI patients.

## 1. Introduction

Sepsis is a life-threatening organ dysfunction resulting from a dysregulation of the body's response to infection [1]. The incidence of sepsis and death rates remain high despite advances in anti-infective treatment and basic life support. One of the most common organs injured in sepsis is the kidney, resulting in sepsis-associated acute kidney injury (SA-AKI) [2]. AKI can occur in 30% to 50% of patients with sepsis in the intensive care unit, which is significantly higher than AKI caused by other causes [3]. In a US study including 192,980 patients with sepsis, 22% of patients with sepsis progressed to AKI, with a 38.2% mortality rate [4]. A multicenter prospective study with 1255 patients found that the incidence of AKI in the ICU was 31.6%, with sepsis accounting for 44.9% of patients [5]. Early diagnosis and timely intervention can improve the prognosis of invalids with SA-AKI [2]. KDIGO defines the diagnosis of SA-AKI more finely, relying on increased serum creatinine or decreased urine output, both of which have their limitations. Because kidney function is highly compensatory, even if one kidney is damaged, the change in serum creatinine level does not fluctuate much. The measurement of urine volume is strongly influenced by the subjectivity of the tester. In order to detect the occurrence of SA-AKI, it is necessary to investigate additional early and efficient biomarkers. However, these markers are currently not used in clinical therapy. Various novel markers may be useful for the early detection of SA-AKI in sepsis.

Noncoding RNAs called miRNAs, which have 21–25 nucleotides, recognise particular target mRNAs and control gene expression. miRNA is crucial in a number of pathogenic processes and can be involved in controlling cell growth, differentiation, metabolism, apoptosis, and other processes [6]. Various miRNAs are involved in the occurrence and development of SA-AKI through different mechanisms such as oxidative stress, inflammatory response, and mitochondrial autophagy [7, 8]. In SA-AKI patient sera, miR-22-3p expression was decreased and was inversely associated with the levels of renal damage markers. miR-22-3p was also useful for diagnosing SA-AKI in patients [9]. There are, however, not many research on the connection between miRNAs and SA-AKI. There are, however, not many miRNAs currently available for the diagnosis of AKI, and there have not been many investigations on the connection between miRNA and SA-AKI. Therefore, more investigation into novel biomarkers for SA-AKI diagnosis and prognosis is required. This study mainly investigated the value of miR-370-3p and miR-495-3p in the noninvasive diagnosis of SA-AKI.

The remaining of this manuscript was arranged as the following: part 2 introduced the basic theory of materials and methods. The third part verified the proposed method through experiments and analyzes the experimental results. Part 4 was conclusion.

## 2. Material and Methods

In this study, 184 sepsis patients were divided two group according to whether they had acute kidney injury, including non-AKI and AKI group. The criteria for defining AKI were as described by Zhang et al. [9]. The patients were excluded in case they (1) aged ≥ 18 years without other major comorbidities and (2) consent to include their own clinical information in this study. Exclusion criteria: (1) patients have other causes of acute kidney injury, including obstruction of the urinary tract system, glomerular necrosis, glomerulonephritis, and nephrovascular disease; (2) myolysis and amputation; and (3) kidney transplantation. The fundamental statistics and clinical details of the patients were summarized in Table 1. On the first day of admission, clinical records for patients are questioned. The experimental project was disclosed to the patients.

### 2.1. Sample Collection

Urine was collected from non-AKI and AKI patients. The specimen was centrifuged at 3000 r/min to obtain the supernatant. Scr and Cys-C concentrations were detected by AU5800 machine (Beckman, USA). NGAL and KIM-1 concentrations were measured via ELISA kits (Absin, China).

### 2.2. RT-qPCR

Total RNA was extracted by Trizol (Absin, China). The RNA of qualified purity was reverse transcribed to cDNA. The real-time PCR reaction was performed using a 7500 PCR instrument (ABI, USA) and SYBR Green kit (Takara, Japan). The primers were designed and synthesized by Tingske Biotech (Table 2).

### 2.3. Follow-Up

Patients diagnosed with SA-AKI need to be followed up for 28 days to record survival and time to death for use in survival curve plotting.

### 2.4. Statistical Analysis

The SPSS 23.0 software was utilized. *T*-test or Chi square test was utilized to compare difference between groups. *P* < 0.05 meant significantly difference. ROC curve was established for measuring the diagnostic value of miR-370-3p and miR-495-3p for SA-AKI. Prediction of SA-AKI prognosis by miR-370-3p and miR-495-3p expression levels was constructed by survival curves.

## 3. Results

### 3.1. Patient Clinical Information

Table 1 displayed the clinical data of the patients. CRP, Scr, Cys-C, NGAL, and KIM-1 were clearly higher in the AKI group compared to non-AKI patients. By comparison with non-AKI patients, PCT was markedly increased in AKI group. There was no difference between the two groups at other indicators.

miR-370-3p and miR-495-3p were lower expressed in SA-AKI patients.

As shown in Figure 1(a), miR-370-3p expression was markedly declined in AKI invalids. In addition, miR-495-3p expression was also markedly declined in sepsis AKI invalids (Figure 1(b)).

### 3.2. Relationship between miR-370-3p, miR-495-3p Expression, and Biomarkers of SA-AKI

Urinary miR-370-3p was significantly correlated negatively with Scr, Cys-C, NGAL, and KIM-1, according to Pearson correlation analysis (Table 3). Similar to the above results, miR-495-3p also showed a significant negative correlation with Scr, Cys-C, NGAL, and KIM-1 (Table 3).

### 3.3. Diagnostic Performance of miR-370-3p and miR-495-3p for SA-AKI

ROC curve was established for measuring the diagnostic value of miR-370-3p and miR-495-3p for SA-AKI. The area under the curve (AUC) of miR-370-3p for diagnosing sepsis AKI was 0.896 (Figure 2(a)). The AUC of miR-495-3p for diagnosing SA-AKI was 0.814 (Figure 2(b)).

### 3.4. Prediction of SA-AKI Prognosis by miR-370-3p and miR-495-3p Expression Levels

Survival curves were constructed to evaluate association between miR-370-3p, miR-495-3p, and patients' 28-day survival. The 28-day survival rate of invalids with high expression of miR-370-3p was obviously higher in contrast to those with lower miR-370-3p expression (Figure 3(a)). Patients with high miR-495-3p expression had significantly higher 28 days-survival rates in contrast to those with low miR-495-3p expression (Figure 3(b)).

## 4. Discussion

A frequent and serious illness known as AKI occurs when kidney function rapidly declines for a variety of reasons. It is a typical critical sickness affecting a number of organs and systems. Acute onset and a significant inflammatory response are the hallmarks of SA-AKI [2]. Patients with SA-AKI have markedly elevated serum creatinine, abnormal liver function, coagulation abnormalities, increased inflammatory markers, hyperuricemia, hyperglycemia, and hyperlactatemia [10], and most patients require hemodynamic support and mechanical ventilation [11]. SA-AKI has a poor clinical prognosis, and the in-hospital mortality rate was approximately 30-50% [12].

The primary diagnostic tool for SA-AKI and an indicator of its severity is currently serum creatinine [13]. However, there are several drawbacks to using serum creatinine as an early SA-AKI diagnosis. First, exogenous creatinine and endogenous creatinine make up creatinine. Consumption of meat-based foods has a direct impact on exogenous creatinine, but endogenous creatinine is influenced by factors such as age, gender, race, exercise, weight, muscle content, and the body's inflammatory response [14]. Second, the kidney is powerful in compensation, and it can maintain the normal value of serum creatinine level even when the unilateral kidney function is functioning [3], and the serum creatinine can be maintained in the normal range in early and mild kidney injury [13]. In addition, urine volume is insensitive to the diagnosis of acute kidney injury and cannot be easily measured outside of the monitoring room. The measurement of urine volume is susceptible to subjective influence. The measurement of urine volume is subjective. Therefore, there is a clinical need for more effective early diagnosis of SA-AKI. Khawaja et al. measured early plasma NGAL concentration in 48 septic patients and found that early NGAL concentration could effectively predict AKI, with AUC of 0.82, sensitivity of 70.8%, and specificity of 90.9%, and NGAL concentration was positively correlated with ICU stay [15].

miRNAs are evolutionarily highly conserved and can regulate gene expression, participating in a variety of pathological and physiological processes [16]. Urine specimens are readily available, and a variety of miRNAs can be detected in urine [17]. miRNAs may reflect the extent of renal tissue damage [18, 19]. The mechanism of miRNA action in SA-AKI has not been elucidated and may contribute to the development of SA-AKI in sepsis patients through ischemia-reperfusion injury, inflammatory mediator release, oxidative stress, and mitochondrial damage. miR-370-3p was lower expressed in SA-AKI patients, and miR-370-3p overexpression could inhibit SA-AKI via targeting MYD88 [20]. miR-495-3p was reported to be regulated by SNHG14 to alleviate SA-AKI and lower expressed in SA-AKI patients [21]. In the current investigation, sepsis AKI patients' urine miR-370-3p and miR-495-3p expression levels were significantly lower than those of non-AKI patients. These findings showed that miR-370-3p and miR-495-3p may serve as novel biomarkers for SA-AKI.

Next, we further explored the association of miR-370-3p and miR-495-3p with known AKI biomarkers. Pearson correlation analysis demonstrated miR-370-3p and miR-495-3p were markedly negatively correlated with AKI biomarkers. In addition, ROC curve was established for measuring diagnostic value of miR-370-3p and miR-495-3p for SA-AKI. The AUC of miR-370-3p and miR-495-3p for diagnosing sepsis SA-AKI was 0.896 and 0.814, respectively. These results demonstrated miR-370-3p and miR-495-3p were useful for the diagnosis of SA-AKI. The 28-day survival rate of invalids with high expression of miR-370-3p was obviously higher in contrast to those with lower miR-370-3p expression. Patients with high miR-495-3p expression had significantly higher 28 days-survival rates in contrast to those with low miR-495-3p expression.

In conclusion, the current investigation showed that miR-370-3p and miR-495-3p in the urine were involved in the diagnosis of SA-AKI, and the procedure is quick, easy, safe, and noninvasive. However, there are few studies on miR-370-3p and miR-495-3p and AKI, especially SA-AKI. The role of miR-370-3p and miR-495-3p in SA-AKI needs to be confirmed by further studies.

## Figures and Tables

**Figure 1:** Urinary miR-370-3p (a) and miR-495-3p (b) expressions were measured by RT-qPCR for sepsis AKI.

**Figure 2:** ROC curve analysis of urinary miR-370-3p (a) and miR-495-3p (b) for SA-AKI.

**Figure 3:** Kaplan-Meier survival analysis of 28 d survival rate according to urinary miR-370-3p (a) and miR-495-3p (b) levels.

**Table 1:** Patient clinical information.

Items	Non-AKI (*n* = 49)	AKI (*n* = 39)	*P*
Age (years)	51.23 ± 9.76	49.77 ± 9.960	0.318
Gender (male/female)	56/40	48/40	0.605
BMI (kg/m^2^)	20.87 ± 2.41	21.08 ± 2.290	0.543
Hypertension	21	17	0.669
Diabetes mellitus	10	12	0.501
Cardiovascular disease	7	4	0.433
CRP (ng/mL)	65.27 ± 24.860	83.92 ± 31.630	0.001
PCT (ng/mL)	3.94 ± 0.990	3.47 ± 1.570	0.014
WBC (×10^9^/L)	14.86 ± 6.390	15.77 ± 8.270	0.403
eGRF (mL/min per 1.73 m^2^)	61.76 ± 14.540	49.91 ± 18.570	<0.001
Scr (*μ*M)	94.39 ± 27.020	151.79 ± 28.050	<0.001
Cys-C (mg/L)	0.58 ± 0.090	2.10 ± 0.460	<0.001
NGAL (ng/mL)	53.36 ± 15.110	80.38 ± 17.980	<0.001
KIM-1 (ng/mL)	4.55 ± 0.460	21.81 ± 5.550	<0.001

**Table 2:** Primer sequences.

Items	Primer sequences (5′-3′)
miR-370-3p	F:GCCTGCTGGGGTGGAACCTGGT
	R:CTCAACTGGTGTCGTGGA
miR-495-3p	F: AAACAAACATGGTGCA
	R: GAGCAGGCTGGAGAA
*β*-Actin	F:GCACCACACCTTCTACAATG
	R:TGCTTGCTGATCCACATCTG

**Table 3:** Correlation between miR-370-3p, miR-495-3p, and SA-AKI biomarkers.

Items	miR-370-3p		miR-495-3p	
	*r* value	*P* value	*r* value	*P* value
Scr (*μ*M)	-0.661	0.001	-0.564	0.001
Cys-C (mg/L)	-0.615	0.001	-0.478	0.001
NGAL (ng/mL)	-0.714	0.001	-0.596	0.001
KIM-1 (ng/mL)	-0.623	0.001	-0.514	0.001

## Data Availability

Data to support the findings of this study is available on reasonable request from the corresponding author.
